This article has been retracted.

# Mechanistic modeling and numerical simulation of axial flow catalytic reactor for naphtha reforming unit

**DOI:** 10.1371/journal.pone.0242343

**Published:** 2020-11-20

**Authors:** Mahboubeh Pishnamazi, Ali Taghvaie Nakhjiri, Mashallah Rezakazemi, Azam Marjani, Saeed Shirazian

**Affiliations:** 1 Institute of Research and Development, Duy Tan University, Da Nang, Vietnam; 2 The Faculty of Pharmacy, Duy Tan University, Da Nang, Vietnam; 3 Department of Petroleum and Chemical Engineering, Science and Research Branch, Islamic Azad University, Tehran, Iran; 4 Faculty of Chemical and Materials Engineering, Shahrood University of Technology, Shahrood, Iran; 5 Department for Management of Science and Technology Development, Ton Duc Thang University, Ho Chi Minh City, Vietnam; 6 Faculty of Applied Sciences, Ton Duc Thang University, Ho Chi Minh City, Vietnam; 7 Laboratory of Computational Modeling of Drugs, South Ural State University, Chelyabinsk, Russia; Universiti Malaysia Pahang, MALAYSIA

## Abstract

Naphtha catalytic reforming (NCR) process has been of tremendous attention all over the world owing to the significant requirement for high-quality gasoline. Industrialized naphtha reforming unit at oil refineries applies a series of fixed bed reactors (FBRs) to improve the quality of the low-octane hydrocarbons and convert them to more valuable products. The prominent purpose of this research is to understand the catalytic reactor of naphtha reforming unit. For this aim, an appropriate mechanistic modeling and its related CFD-based computational simulation is presented to predict the behavior of the system when the reactors are of the axial flow type. Also, the triangular meshing technique (TMT) is performed in this paper due to its brilliant ability to analyze the results of model’s predictions along with improving the computational accuracy. Additionally, mesh independence analysis is done to find the optimum number of meshes needed for reaching the results convergence. Moreover, suitable kinetic and thermodynamic equations are derived based on Smith model to describe the NCR process. The results proved that the proceeding of NCR process inside the reactor significantly increased the concentration amount of aromatic materials, lighter ends and hydrogen, while deteriorated the concentration amount of naphthene and paraffin. Moreover, the pressure drop along the reactor length was achieved very low, which can be considered as one of the momentous advantages of NCR process.

## 1. Introduction

It is known that naphtha is one of the most important intermediate products of crude oil refining industry. This product is extensively applied as feed in petroleum refining units such as steam cracking, catalytic reforming, and isomerization [1]. Naphtha consists of hydrocarbons containing 5 to 12 carbon atoms with boiling points ranging from 30 to 200°C. It means that if the crude oil is heated in the temperature range of 30 to 200°C and the boiled part is separated, naphtha would be obtained. Usually, 15 to 30% of crude oil boils at this temperature, so the same amount of crude oil can be converted directly to naphtha [2, 3].

The catalytic reforming process of naphtha has been developed rapidly over the past four decades and has become one of the most advanced units in the refining industry. The prominent aim of this process is to convert low octane hydrocarbons to high octane reforming products for application as efficient fuel. Hydrogen and other light gases (i.e. propane and butane) are considered as the byproducts of the aforementioned process [1, 4]. For optimal results of the catalytic reforming process, catalyst, computational fluid dynamics (CFD), and process technology should be taken into account and combined [5]. Process engineers and catalyst manufacturers are trying to present different ways to improve process efficiency and catalyst selectivity toward increased production of aromatics and high-octane reforming products [6].

The reforming feed is composed of various paraffinic, naphthenic, aromatic, and rarely olefinic hydrocarbons containing 5 to 10 carbons. There are two types of feed for the naphtha catalytic reforming (NCR) unit [1, 7]:

1. Naphthenic feed that has a high total amount of naphthene and aromatic compounds.
2. Paraffinic feed with a higher percentage of paraffinic compounds.

The naphthenic feed can produce a product with a higher octane number in milder conditions in terms of temperature and operating pressure because it has a high percentage of naphthenic compounds and the conversion of naphthene to aromatic compounds (compounds with high octane, which is the main factor in raising octane number of gasoline) is done very quickly and does not require harsh operating conditions [1, 7].

CFD is appropriately perceived as a trustworthy procedure to model the refining processes such as NCR and analyzing their corresponding momentum and mass transport equations [8, 9]. In this paper, COMSOL is applied as the governing software to provide a computational simulation for the radial flow catalytic reactor of the naphtha reforming unit. The existence of outstanding abilities such as accuracy, simplicity of application, and robustness has persuaded the investigators to apply this technique compared to other commercial software [10–13]. Mostafazadeh et al. theoretically investigated the efficiency, optimum operating conditions, and increment of the aromatic production in a Pd–Ad membrane reactor for the NCR process. They found that the hydrogen permeation through the membrane eventuated in changing the reaction direction towards the product side based on the thermodynamic equilibrium [14]. Hu et al. proposed molecular modeling and process optimization for the NCR unit. They perceived that increment in temperature would be able to improve the Research Octane Number (RON) for the gasoline and enhanced benzene and aromatics. While increasing the temperature negatively affected the recovery ratio of stabilizing gasoline, which generally deteriorated the profit [15].

This work aimed to propose a mathematical modeling and its related CFD-based computational simulation to prognosticate the behavior of the NCR's reactors when they are of the axial flow type. To do this, COMSOL software is applied due to its capabilities (i.e. ease of use and accuracy) to analyze and solve mass and momentum transport equations. Moreover, the study on the concentration variations of desired components such as naphthene, aromatic materials, hydrogen, lighter ends, and paraffin along the length of the NCR reactor and the change of temperature and pressure inside the reactor is another objective of this study.

## 2. Model development

Experiments have shown that naphtha is composed of more than three hundred different compounds with different physico-chemical properties. These compounds are mainly composed of naphthenes, paraffins and aromatics, which undergo various reactions. Numerous kinetic models have been proposed to illustrate the main compounds and reactions involved in the NCR reaction. One of the simplest and at the same time, efficient models is the Smith model. The naphtha feed is significantly complex including numerous components that each of them undergoes different reactions. The development of an appropriate model propounding all the components/reactions is believed to be complex. Therefore a suitable lumping of the components using carbon number based on similar properties and kinetic behavior might be more efficient. Smith worked on developing a model pondering naphtha as naphthenes, paraffins, and aromatics lump with average carbon number properties. In this model, the reactions in NCR process are divided into four main reactions, which are as follows [6]:

1. Dehydrogenation of naphthenes to aromatics:
  $$N(C_{n}H_{2n})⇌A(C_{n}H_{2n-6})+3H_{2}$$ (1)
2. Dihydrocyclization of paraffins to naphthenes:
  $$N(C_{n}H_{2n})+H_{2}⇌P(C_{n}H_{2n+2})$$ (2)
3. Hydrocracking of naphthenes:
  $$N(C_{n}H_{2n})+\frac{n}{3}H_{2}⇌Lighter\;ends(C_{1}-C_{5})$$ (3)
4. Hydrocracking of paraffins:
  $$P(C_{n}H_{2n+2})+\frac{n-3}{3}H_{2}⇌Lighter\;ends(C_{1}-C_{5})$$ (4)

The reaction rates of the above-mentioned equations can be expressed by applying the following equations [6]:

$$r_{1}=\left(\frac{k_{f1}}{K_{e1}}\right)(k_{e1}p_{n}-p_{a}p_{h}^{3})$$ (5)

$$r_{2}=\left(\frac{k_{f2}}{K_{e2}}\right)(k_{e2}p_{n}p_{h}-p_{p})$$ (6)

$$r_{3}=\left(\frac{k_{f3}}{p_{t}}\right)p_{n}$$ (7)

$$r_{4}=\left(\frac{k_{f4}}{p_{t}}\right)p_{p}$$ (8)

where *k*_*fi*_, *K*_*ei*_, and *p*_*i*_ denote the reaction rate constants, equilibrium constants, and partial pressure of components *i* (i.e., aromatics, naphthenes, paraffins and hydrogen), respectively. The rate constants required to calculate the equilibrium constants are presented in Table 1 where *E*_*i*_ and Δ*H*_298*K*_ are expressed as the activation energies and standard heat of reaction, respectively [16].

**Table 1:** Heat of reactions and rate constants for NCR process [16].

$k=A\;exp\;(B-\frac{E}{1.8T})$	ΔH_298K_	E	B	A
*k*_*f*1_	71038.06	30630	21.4	9.87
*k*_*f*2_	-36953.33	51670	32.54	9.87
*k*_*f*3_	-51939.31	57211	39.54	1
*kf*_4_	-56597.54	57211	39.45	1
*K*_*e*1_	--	50580	54	1040
*K*_*e*2_	--	9150	-9.43	9.87

Mathematical modeling of these catalytic reactors has been developed by deriving mass and energy balance equations and considering the following assumptions:

1. Steady-state condition is considered to develop the mechanistic model;
2. The developed model is homogeneous;
3. The ideal gases law is applied for the compounds present in the process (due to low pressure and high temperature)

Derivation of the mass balance and combining the kinetic and thermodynamic equations eventuates in the achievement of the concentration distribution equations of naphthenes, aromatics, paraffins and hydrogen in different radial positions of catalytic reactor. From the enthalpy balance and the combination of the same kinetic and thermodynamic equations, the equation of temperature distribution in the reactor is obtained. The equations related to the mass balance of all the chemical components involved in the reaction for the porous catalytic reactor are as follows [17–22]:

$$u\nabla .C_{i}=\nabla .(D_{i}\nabla .C_{i})+r_{i}$$ (9)

$$N_{i}=-D_{i}\nabla .C_{i}+u\nabla C_{i}$$ (10)

where *N*_*i*_, *C*_*i*_, *r*_*i*_ and *D*_*i*_ are denoted as the flux, concentration, reaction rate, and diffusion coefficients of components i (aromatics, naphthenes, paraffins, hydrogen and lighter ends) involved in the reaction of NCR process. The reaction rate for naphthenes, aromatics, paraffins, and hydrogen participating in the reaction is as follows [18, 23]:

$$r_{A}=\rho_{b}.r_{1}$$ (11)

$$r_{N}=\rho_{b}.(-r_{1}-r_{2}-r_{3})$$ (12)

$$r_{P}=\rho_{b}.(r_{2}-r_{4})$$ (13)

$$r_{H}=\rho_{b}.\left(3r_{1}-r_{2}-\frac{n-3}{3}r_{4}-\frac{n}{3}r_{3}\right)$$ (14)

$$r_{L}=\rho_{b}.\left(\frac{n-3}{3}r_{4}+\frac{n}{3}r_{3}\right)$$ (15)

where *ρ*_*b*_ is expressed as the reactor bulk density. The equations related to the fluid energy balance for the porous catalytic porous reactor are as follows [24–26]:

$$\rho C_{P}u.\nabla T=\nabla .(k\nabla T)+Q$$ (16)

$$\rho C_{P}u.\nabla T=\nabla .(k_{eff}\nabla T)+Q$$ (17)

$$k_{eff}=\theta_{p}k_{p}+(1-\theta_{p})k$$ (18)

where *C*_*P*_, *u*, *Q*, *k*_*eff*_, *θ*_*p*_ and *k*_*p*_ are interpreted as the specific heat capacity, velocity, volumetric flow rate, effective thermal conductivity, porosity, and thermal conductivity of the porous reactor, respectively. The momentum equations related to the fluid motion for a porous catalytic reactor can be presented as follows [24–26]:

$$r_{A}=\rho_{b}.r_{1}$$ (19)

$$\rho (u.\nabla )u=\nabla .\left(-pl+\mu (\nabla u+{(\nabla u)}^{T})\right)+F$$ (20)

ρ∇.u=0 (21)

$$\frac{\rho }{\epsilon_{p}}\left((u.\nabla )\frac{u}{\epsilon_{p}}\right)=\nabla .\left[-pl+\frac{\mu }{\epsilon_{p}}(\nabla u+{\left(\nabla u\right)}^{T})-\frac{2\mu }{3\epsilon_{p}}(\nabla u)l\right]-\left(\mu \kappa^{-1}+\beta_{F}|u|+\frac{Q_{br}}{\epsilon_{p}^{2}}\right)u+F$$ (22)

$$\rho \nabla .u=Q_{br}$$ (23)

where viscosity, velocity vector, body force term, pressure, fluid density, permeability and porosity are respectively expressed as *μ*, *u*, *F*, *p*, *ρ*, *κ* and *ϵ*_*p*_, respectively. The required physical variables/parameters to develop the mathematical modeling and computational simulations are listed in Table 2.

**Table 2:** Required parameters for model development.

Parameter	Unit	Value	Ref.
Diameter of reactor (D)	m	1.25	[18]
Reactor length (L)	m	6.29	[18]
Cross section (A_c_)	m^2^	1.2272	Calculated from [18]
Fluid viscosity (μ)	mPa.s	0.01	[18]
Fluid velocity (u_0_)	m/s	0.58	[18]
Fluid density (ρ_f_)	kg/m^3^	14.904	[18]
Specific heat capacity (C_pf_)	J/(kg.K)	3384.6	[18]
Temperature (T_i_)	K	777	[18]
Pressure (P_i_)	kPa	P_total_	[18]
P_total_	kPa	3703	[18]
Volumetric flow rate (Q)	m^3^/s	0.71177	[18]
Porosity of catalyst (ε)	--	0.36	[18]
Specific surface (A_s_)	m^2^	3.29	[18]
Diameter of catalytic particles (d_p_)	m	4.7×10^−3^	[18]
Mole fraction of naphtha (x_n_)	--	0.0461	[18, 27]
Mole fraction of paraffin (x_p_)	--	0.0631	[18, 27]
Mole fraction of aromatics (x_a_)	--	0.0188	[18, 27]
Mole fraction of lighter components (x_l_)	--	0.266	[18, 27]
Mole fraction of hydrogen (x_h_)	--	0.606	[18, 27]
Naphtha concentration (c_n_)	mol/m^3^	26.462	Calculated from [18, 27]
Paraffin concentration (c_p_)	mol/m^3^	36.17	Calculated from [18, 27]
Aromatics concentration (ca)	mol/m^3^	10.777	Calculated from [18, 27]
Hydrogen concentration (c_h_)	mol/m^3^	347.37	Calculated from [18, 27]
Lighter components concentration (c_l_)	mol/m^3^	152.48	Calculated from [18, 27]

In this investigation, triangular meshing technique (TMT) is implemented due to its momentous capability to analyze the results of model’s predictions along with increasing the computational accuracy. TMT can divide the entire geometry of NCR reactor into a very small dimension and cover all of the dead zones inside it, which results in enhancing the precision of the developed model. It is worth mentioning that the density and size of meshes in the proximity of the boundary walls are remarkably higher and finer, respectively, which results in improving the precision of model results and minimizing the computational errors. Fig 1 illustrates the triangular meshing in the domain of the catalytic reactor.

**Fig 1:** Implemented TMT inside the domain of catalytic reactor.

To investigate the mesh independence, it is essential to mention that although enhancement in the number of meshes eventuates in decreasing the computational errors and simultaneously improving the precision of model predictions, it also considerably increases the computational time. Hence, it seems to be essential to achieve an optimum number of meshes for the numerical simulations of process. The effect of mesh numbers on the amount of naphthene concentration at the outlet of the NCR reactor is depicted in Table 3. It is perceived from the Table 3 that enhancement in the number of meshes results in variations of naphthene concentration, but, after the 360th mesh, no substantial alterations in the amount of naphthene concentration at the outlet of the NCR reactor takes place, which implies adequacy of the meshes number after the 360th mesh and convergence of results. Therefore, the computational precision of the model predictions is independent of the number of meshes after 360th mesh, and hereafter this number is considered for further investigations.

**Table 3:** The influence of mesh numbers on the amount of naphthene concentration at the outlet of the NCR reactor.

Number of mesh	Naphthene concentration at the outlet of the NCR reactor
60	9.70
120	10.25
180	10.50
240	10.80
300	11.00
360	11.197
420	11.198
480	11.199
540	11.20

## 3. Results and discussion

### 3.1 Model validation

The validation of model predictions has been performed via comparison of plant data for normally packed bed reactor (NPBR) considering steady-state circumstances. As demonstrated in Table 4, an excellent agreement exists between the outlet temperature of plant and NPB reactor with the average relative deviation (ARD) of about 0.13%, which corroborates the validation of model results.

**Table 4:** Comparison of model prediction and plant data.

Number of Reactor	Outlet temperature of Plant (K)	Outlet temperature of NPBR (Model prediction) (K)	ARD (%)
1	722	723	0.13

### 3.2 Concentration profile of naphthene and aromatics inside the catalytic reactor

NCR process is known as the most prominent industrial operation applied by petroleum refineries to convert paraffins and naphthenes into aromatic (2). Naphthenic compounds are converted to aromatic materials during the dehydrogenation reaction. These compounds are also converted to lighter ends (lighter products) under the hydrocracking reaction. Fig 2A and 2B present the concentration profile of naphthene and aromatics inside the catalytic reactor of NCR process. As shown in Fig 2A, the amount of naphthenic compounds decreases substantially from 26.4 to 11.2 mol.m^-3^ along the length of the catalytic reactor due to their consumption in dehydrogenation and hydrocracking reactions. It should be noted that despite the production of naphthenic products in the dihydrocyclization reaction, due to the predominance of two naphthenic reactions (dehydrogenation and hydrocracking), which consume naphthenic compounds, the molar flow of these compounds decreases along the length of the catalytic reactor. The purpose of the naphtha reforming reaction is to produce aromatic compounds that have a high octane number. In this reaction, paraffinic and naphthenic compounds are converted to aromatics, so the amount of aromatics increases continuously throughout the reactor. The concentration of aromatic materials along the reactor length is shown in Fig 2B.

**Fig 2:** Concentration profile of a) naphthene and b) aromatic materials inside the NCR reactor.

### 3.3 Concentration profile of lighter ends along the reactor length

The light gases contain light by-products (lighter ends) that are mainly produced by the hydrocracking reaction during the NCR process. These materials are used as feed in the production of liquefied petroleum gas (LPG). Fig 3 shows the concentration profile of lighter ends along the reactor length. Accordingly, the increasing trend of lighter ends production during the reactor is shown, which can be attributed due to increasing the durability of the hydrocracking reaction inside the NCR reactor.

**Fig 3:** Concentration gradient of lighter ends along the length of NCR reactor.

### 3.4 Pressure and temperature profiles along the NCR reactor length

Fig 4 illustrates the temperature profile along the reactor length. Because of the significantly endothermic characteristics of the important reforming reactions, temperature declines by progressing the reactions, which eventuates in considerable deterioration in the production rate. Therefore, to keep the temperature of reaction at an appropriate level, industrial catalytic reformers are designed to possess multiple reactors and intermediate furnaces. Fig 5 depicts the pressure profile inside the NCR reactor. One of the momentous privileges of the NCR is the existence of insignificant pressure loss inside the reactors, which permits the application of smaller particles of the catalyst with superior efficiency. As observed, the pressure change through the reactor is low and sudden decline is seen during a stream passage through one reactor to another because of piping/instruments.

**Fig 4:** Temperature profile along the NCR reactor length.

**Fig 5:** Pressure profile inside the NCR reactor.

### 3.5 Concentration profiles of hydrogen and paraffin along the NCR reactor

Figs 6 and 7 illustrate the concentration profiles of hydrogen and paraffin along the NCR reactor. Hydrogen is appropriately perceived as one of the important by-products of the NCR process. By proceeding the NCR process inside the reactor, hydrogen is produced during the dehydrogenation reaction of naphthenes to aromatics, while this by-product is consumed in the other reactions of NCR process, including dihydrocyclization of paraffin to naphthenes, hydrocracking of naphthenes and hydrocracking of paraffins. Due to the predominance of H_2_ production in dehydrogenation reaction of naphthenes than the reactions produce hydrogen, the amount of hydrogen concentration along the reactor length increases from 348 to 387 mol m^-3^. According to Smith's kinetic model, paraffins are converted to naphthenes under the dihydrocyclization reaction. These compounds also undergo the hydrocracking reaction and are converted to lighter compounds. Therefore, as shown in Fig 7, the amount of paraffinic materials decreases along the reactor length.

**Fig 6:** Concentration profiles of hydrogen along the reactor length.

**Fig 7:** Concentration profiles of paraffin along the reactor length.

## 4. Conclusions

In this study, a mechanistic modeling and its related CFD-based simulation was developed to investigate the catalytic reactor of naphtha reforming unit. The results corroborated the accuracy of the kinetic equations used for this model. The developed model can be applied to predict the amount of aromatic capacity, process efficiency, transfer rate, bed temperature and finally system conditions in case of changes in operating conditions. Some important parameters such as reaction temperature/pressure considerably affect the efficiency of the NCR process. Therefore, variations of temperature and pressure along the axial coordinate (length) of reactor and also the variations of desired components concentration such as naphthene, aromatic materials, hydrogen, lighter ends and paraffin along the length of NCR reactor have been evaluated. Based on the results, substantial endothermic behaviour of the important reforming reactions caused the decrement in the temperature inside the reactor while the pressure drop along the reactor length was insignificant, which facilitates the application of smaller catalyst particles.
